# Significant Association of rs2147555 Genetic Polymorphism in the *EDNRB* Gene with Hirschsprung Disease in Southern Chinese Children

**DOI:** 10.1155/2020/5956412

**Published:** 2020-10-31

**Authors:** Yi Zheng, ChaoTing Lan, Ning Wang, Xiaogang Xu, Tuqun Hu, Qi Wu, Xiaoli Xie, Zhe Wang, Yan Zhang, Cong Li

**Affiliations:** Department of Pediatric Surgery, Guangdong Provincial Key Laboratory of Research in Structural Birth Defect Disease, Guangzhou Women and Children's Medical Center, Guangzhou Medical University, Guangzhou, 510623 Guangdong, China

## Abstract

Hirschsprung disease (HSCR) is a human birth defect at the clinical setting, usually characterized by an absent enteric nervous system (ENS) from the distal bowel. The majority of HSCR cases represent a complex disorder resulting from the interaction of multiple genetic and environmental factors. Genetic events have been described to be involved in the abnormal development of the enteric nervous system. Although variants in several genes like *RET* and *EDNRB* have been suggested to contribute major risks to HSCR, very little is known about their involvement in the onset of HSCR. Here, we studied a large Chinese Han cohort consisting of 1,470 HSCR patients and 1,473 non-HSCR controls to further test whether there are more variants in *EDNRB* associated with HSCR. Our results provided the first evidence that rs2147555 in *EDNRB* confers a significant risk of HSCR in a Chinese Han population for both allelic frequencies (*P* = 4.16 × 10^−3^; OR = 1.29) and genotypic frequencies assuming either a dominant or recessive model (*P* = 0.011 and *P* = 0.027, respectively). When different subtypes of HSCR cases were analyzed, the association remained significant (OR = 1.33, *P* = 0.003 for short-segment HSCR; OR = 1.34, *P* = 0.044 for long segment HSCR).

## 1. Introduction

Hirschsprung's disease (HSCR) is a common birth defect in clinical practice characterized by disturbed development of ENS due to abnormal differentiation or survival of the enteric neural crest-derived cells (ENCCs). Patients with HSCR usually have continued bowel dysfunction including colonic obstruction, constipation, and enterocolitis [1]. HSCR has an estimated prevalence rate of around 2.8 cases per 10,000 live births in Asia, with a male/female ratio of approximately 4 : 1 [2]. Based on varying lengths of aganglionosis, at least 3 subtypes of HSCR have been reported: long-segment HSCR (L-HSCR), short-segment HSCR (S-HSCR), and total colonic aganglionosis (TCA). In addition, rare cases with the aganglionosis extending to the small bowel (total intestinal aganglionosis (TIA)) are the most severe form of HSCR and are often lethal [3, 4].

Genetic risk factors are very likely to play an important role in the pathogenesis of HSCR, although HSCR is a non-Mendelian, multigenic disease. Most of the HSCR cases are sporadic, but some cases have been found to occur in families (5%~20%) [5]. In recent years, genetic studies have led to the discovery of genes that are expressed in the ENS and are involved in the early differentiation of ENCCs into enteric neurons, chiefly the genes encoding the *RET*/*GFRα1*/*GDNF* pathway and the *EDNRB*/*EDN3* pathway [6, 7]. The protooncogene *RET* is a member of the receptor tyrosine kinase family of proteins, and variants of *RET* have been identified in patients with several types of cancer. It has been estimated that variants of *RET* contribute to about 20% of all HSCR cases, most of which can lead to insufficient doses or loss of function of the *RET* protein. *RET* is widely known as the main contributor predisposing to HSCR [7–9]. *GFRA1* encodes for the glycosylphosphatidylinositol-linked receptor, which forms a complex with the glial cell line-derived neurotrophic factor (GDNF). GDNF can bind and activate the receptor tyrosine kinase RET; then, it activates downstream pathways. RET and its ligand GDNF both play critical roles for the proliferation, colonization, migration, and differentiation of ENCCs [10].

The *EDNRB*/*EDN3* signaling pathway has been studied in the pathogenesis of HSCR. *EDNRB* encodes for the endothelin receptor B, which activates a phosphatidylinositol-calcium second messenger system, and *EDNRB* is activated during cell proliferation and differentiation. However, the knowledge about its function in ENS is limited. A previous study showed that the blockade of *EDNRB* signaling led to the HSCR phenotype in the enteric neural crest cells (ENCCs) in a mouse model, demonstrating that *EDNRB* and its ligand *EDN3* proteins played pivotal roles in the development and differentiation of ENS [11]. HGMD and ClinVar reported 489 disease-associated variants for HSCR; among them, 42 are located in *EDNRB* and 132 in *RET* [12, 13]. A genome-wide association study (GWAS) carried out in the Mennonite family trios has found out susceptibility loci at *RET*, *EDNRB*, and 16q23, which were observed to be associated with HSCR [14]. Another GWAS study in a Korean HSCR cohort identified SNP rs77743549, which was strongly associated with the length of aganglionosis [15]. So far, more than 20 *EDNRB* variants have been identified in patients with familial and sporadic HSCR, accounting for only 5% of all HSCR patients [16, 17]. Thus, known variants of *RET* and *EDNRB* reported in HSCR explains for the small proportion of HSCR patients indicating that additional variants need to be identified [16].

Previous studies raised the question whether there are more *EDNRB* SNPs, even possibly causal ones, independently associated with HSCR. This made further investigations on this gene of high interest necessary. The molecular mechanism by which *EDNRB* intronic SNPs confer risks on HSCR is not fully understood yet, since most of the SNPs are located in introns; one possibility is that intronic SNPs affect the expression level of *EDNRB* by modulating the regulation of *EDNRB* transcription or pre-mRNA splicing because such regulatory roles have been found for intronic sequences [17]. Moreover, these findings need to be confirmed in a larger population sample and/or in multiple centers. Therefore, we performed a large-scale case-control association study with 1,470 HSCR patients and 1,473 healthy controls in a Chinese Han population to identify more independently associated loci, to explain the complex pattern of inheritance of HSCR, and to further provide the evidence of HSCR susceptibility of the *EDNRB* locus to the variable length of aganglionosis.

## 2. Methods

### 2.1. Study Subjects

The study subjects were selected from a large ongoing Chinese Han database of Guangzhou Women and Children's Medical Center with clinical data and tissue samples of HSCR patients and controls enrolled mainly from southern China. This study was approved by the local ethics committees on human subject research, and informed consent was obtained from guardians of all participants. For HSCR, the study subjects were recruited among individuals who underwent physical examination, radiology, and histological examination of colon biopsies. HSCR was confirmed by experienced pathologists according to the absence of parasympathetic intrinsic ganglion cells in the submucosal and myenteric plexuses. All study participants were of the ethnics of Han origin by self-report. Relevant clinical data were also collected by direct interview or from medical files on age, gender, enteritis, onset month, recurrence status, and subtyping. The control samples were unrelated healthy Han individuals, acquired from pediatric departments of Guangzhou Women and Children's Medical Center who were verified to be free of HSCR based on medical files at the time of enrollment. To minimize the effect of population stratification, the cases matched with controls from the same geographical area.

### 2.2. SNP Genotyping

Human genomic DNA was extracted from venous blood samples of cases and controls using the Wizard® Genomic DNA Purification Kit (Promega Corporation, Madison, WI, USA) following the manufacturer's protocol. Genotyping was performed by using the middle-throughput iPLEX Sequenom MassARRAY platform. Only SNP rs2147555 was selected in our study after filtering; the selection was made according to the Regulome Database. We kept SNPs with high probability to be regulatory variants (RegulomeDB score higher than 2f; https://regulomedb.org/). *EDNRB* SNPs with minor allele frequency (MAF) larger than 5% in the Chinese population (CHB) were also kept (https://www.ncbi.nlm.nih.gov/snp/?term=). Only one SNP was kept if there were two SNPs with a linkage disequilibrium (*r*^2^) larger than 0.8. Two positive controls for each genotype were included in each run. In order to verify the genotyping results, we randomly selected 100 cases and controls for direct DNA Sanger sequencing. The sequencing results for the 100 samples perfectly matched the results of the Sequenom MassARRAY platform.

### 2.3. Statistical Analysis

The SNP genotype was tested for Hardy-Weinberg's equilibrium in the control population using PLINK v1.9. The SNP was assessed for association with HSCR using a comparison of the minor allele frequency in patients and controls, and also other tests (genotypic test of 3 × 2 contingency tables and the tests of dominant or recessive models) using PLINK v1.9. Odds ratios (ORs) and 95% confidence intervals (CIs) were calculated using PLINK v1.9. Logistic regression analysis and empirical *P* value calculation with 100,000 Monte Carlo simulations were carried out by the PLINK v1.9 program. Statistical power was estimated using the Power and Sample Size Program 3.0 assuming an alpha value of 0.05, a two-sided test, and minor allele frequencies for the Chinese population from the 1000 Genomes Project. For our study, our case-control cohort has sufficient power to assess the association between SNPs and HSCR.

## 3. Results

### 3.1. Characteristics of all Participants

We have summarized the general and clinical characteristics of the study cohort in Table 1. A total of 1,470 HSCR cases were selected. The age of onset varied from several days after birth to 14 years old, and the average onset month was 8.37 ± 20.5. A total of 1,473 age-matched healthy controls were recruited from other pediatric departments. A majority of the HSCR cases (70.3%) were classified as S-HSCR, 20.1% and 5.6% were classified as L-HSCR and TCA, respectively, and 3 cases were diagnosed as rare TIA. As the most common postsurgical outcome for HSCR, postsurgery enteritis has similar prevalence of presurgery enteritis in the HSCR group (Table 1).

### 3.2. Association of SNPs with HSCR Risk

SNP rs2147555 was selected for screening to figure out if it was independently associated with HSCR in the South Chinese population. The distribution of three genotypes for SNP rs2147555 was in Hardy-Weinberg's equilibrium in the control group (*P* > 0.05). Significant allelic association was identified between the minor allele C of SNP rs2147555 and HSCR (*P*_obs_ = 4.16 × 10^−3^, OR = 1.291, 95% CI of 1.084-1.538) (Table 2). The association remained significant after adjusting for the covariate of sex which was a risk factor for HSCR (*P*_adj_ = 0.018, Table 2). To better dissect the effective pattern of rs2147555, we have designated 3 different genetic models to the genotypic association, and we found out a significant effect of SNP rs2147555 on HSCR assuming a dominant, recessive, or genotypic model (*P*_obs_ = 0.011, 0.027 and 0.004, respectively). The above association of the different models remained significant with 100,000 Monte Carlo simulations (Table 3).

### 3.3. Stratification Analysis

In the HSCR group, a total of 1034 patients were classified as S-HSCR, accounting for 70.3% of all HSCR cases. Allele C of SNP rs2147555 was notably detected to be associated with S-HSCR (*P*_obs_ = 0.003, OR = 1.33 for allelic frequencies), and rs2147555 genotypes AC/CC were associated with S-HSCR (0.006 for a dominant model, and 0.003 for a genotypic model) (Tables 2 and 3). Allelic association with HSCR remained significant after adjusting for sex (*P*_adj_ = 0.022, Table 2), and dominant and genotypic associations remained significant with Monte Carlo simulation (Table 3). We found marginally significant allelic C association with L-HSCR, and genotypic and recessive models also showed significant associations (Tables 2 and 3). TCA and TIA were both rare and severe HSCR cases, with a proportion of only 5.6% and 0.2%, respectively. No association was found between SNP rs2147555 and TCA/TIA due to a very small number of cases. We carried out Breslow-Day's tests for all of the above stratified associations, but we did not find a significant difference between the ORs for S-HSCR (1.33) and L-HSCR (1.34) (*P* = 0.69).

## 4. Discussion

Many case-control and GWAS studies in Chinese and other races have linked *EDNRB* SNPs to HSCR risk. In this case-control study, we succeeded in identifying the novel intronic SNP rs2147555 in the *EDNRB* gene on chromosome 13q22, which was significantly associated with HSCR in a Southern Chinese population. Our case-control association study has involved 1,470 Chinese HSCR patients and 1,473 non-HSCR controls, all from a large Chinese population of Han ethnic descent. The association between SNP rs2147555 and HSCR was assessed by a 79% power calculated based on the sample size and MAF. For the first time, our group has provided evidence of both allelic and genotypic effects of rs2147555 on the HSCR risk, considering the vital role the EDNRB/EDN3 signaling pathway played in the pathogenesis of HSCR. It is of great significance that the current study has expanded the knowledge of the association of the EDNRB SNPs with the clinical phenotypes of HSCR.

Approximately 70% of HSCR cases were classified as S-HSCR, the most common subtype with missed ENS only in the rectum and sigmoid. 20% of the HSCR cases were classified as L-HSCR, which were more likely to occur in families, suggesting that genetic factors may play a more important role in L-HSCR patients compared to S-HSCR patients. In this study, a significant association of SNP rs2147555 with both S-HSCR and L-HSCR was found, with ORs of 1.33 and 1.34, respectively. The OR for L-HSCR was higher than that for the other subtypes of HSCR, but the difference between ORs was not statistically significant. With respect to other HSCR subtypes, the insufficient number of TCA and TIA cases hampered any conclusion of SNP rs2147555 association. These results demonstrated that the SNP rs2147555 exerted an equal effect in both L-HSCR and “other” HSCR; however, the results needed to be further replicated in other races, considering that the MAF of rs2147555 varied from 0.06 (1000 Genomes-American) to 0.16 (1000 Genomes-African).

We constructed a linkage disequilibrium (LD) map for a 10 kb genomic region including exons 3-6 and part of intron 2 of the *EDNRB* gene and SNP rs2147555 using the genotyping data for the samples of Southern Han Chinese (CHS) and Han Chinese in Beijing (CHB) from the 1000 Genomes Project (hg19) (http://uswest.ensembl.org/Homo_sapiens/Location/LD?r=13:77900000-77910000) (Figure 1). We aimed to find out the possible LD correlation between SNP rs2147555 and exon 3, since rs2147555 and exon 3 of *EDNRB* were only 1.7 kb apart. The LD correlation turned out to be very weak, with an *r*^2^ of 0.11 predicted based on the individuals of the 1000 Genomes CHS data; the *r*^2^ predicted from CHB data was 0 (Figure 1). Therefore, it makes sense to predict that the association of SNP rs2147555 is independent and not due to LD with a potent causative locus in the exons in the population of Southern Han Chinese and also in the Han Chinese in Beijing (mainly Northern Han).

Considerable of evidence has implicated that the *EDNRB*/*EDN3* signaling pathway plays a pivotal role in neural crest-derived cells: ENCC and melanocytes. The *EDNRB* gene encodes for a G-protein-coupled receptor on the migrating ENS precursor surface, and defects in the *EDNRB* gene lead to the blockade of proliferative signals which is needed by ENCCs when they migrate along the bowel. Mutations in the *EDNRB* gene were identified in the Waardenburg syndrome, with clinical pigmentation defects due to abnormal development of melanocytes [18]. A high level of EDNRB can alter precursor differentiation and proliferation then lead to failure of bowel colonization [19]. GWAS studies and replication studies in the Chinese population have identified SNPs in the *EDNRB* gene associated with the risk of HSCR; however, many independent contributors are usually overlooked. Whether these identified SNPs in this region of high interest contribute independent risks to HSCR is still not clear, and validation in a large case-control sample size is necessary. SNP rs2147555 is annotated as a regulatory SNP using RegulomeDB, and the independent effect is also supported by our LD analysis of SNP rs2147555 with the closest coding region of *EDNRB* gene in both north and southern Han Chinese. It is reasonable to hypothesize that rs2147555 may increase the risk of HSCR independently, and future functional investigations will test this hypothesis.

The study has some limitations. First, this is the first time that SNP rs2147555 is found to be associated with HSCR in the Chinese Han population; therefore, the results need to be cross-race validated or further replicated in additional independent Chinese Han populations. Second, environmental factors that may interact with *EDNRB* gene SNPs have not been investigated. Lastly, we cannot exclude selection bias as all the participants were from the same hospital.

In conclusion, the C allele of SNP rs2147555 of *EDNRB* on chromosome 13q22 confers a highly significant risk of HSCR in the Southern Chinese population. The results have expanded the knowledge of association of *EDNRB* SNPs with HSCR previously identified in multiple populations. Nevertheless, future studies with a larger scale of subjects combining genetic and environmental risk factors should be carried out.

## Figures and Tables

**Figure 1:** (a) Overview of linkage disequilibrium (LD) of the 10 kb region around intron 2 of *EDNRB*. The LD structure around SNP rs2147555 was derived from the genotyping data of SNPs from the 1000 Genomes Project Southern Han Chinese (CHS) (http://uswest.ensembl.org/Homo_sapiens/Location/LD?db=core;r=13%3A77900000-77910000). The pairwise correlation between SNPs was measured as *r*^2^, and red refers to *r*^2^ = 1. Exons are marked with yellow boxes. The direction of *EDNRB* transcription is to the left as marked by the arrows. (b) The LD structure between SNP rs2147555 and exons is predicted based on the 1000 Genomes Project for the Han Chinese in Beijing (CHB) population.

**Table 1:** General clinical characteristics of the HSCR case-control cohort.

Characteristic	Cases (*n* = 1,470)	Controls (*n* = 1,473)	*P* ^∗^
Gender (male/female)	1230/240	966/506	0.001
Onset month	8.37 ± 20.5	N/A	—
S-HSCR (%)	1034 (70.3%)	N/A	—
L-HSCR (%)	295 (20.1%)	N/A	—
TCA (%)	82 (5.6%)	N/A	—
TIA (%)	3 (0.2%)	N/A	—
Presurgery enteritis (%)	261 (17.8%)	N/A	—
Postsurgery enteritis (%)	249 (16.9%)	N/A	—

Onset month (mean ± SD): age (month) of onset for HSCR cases; ^∗^*P* is derived from an unpaired Student's *t*-test or Pearson's chi-square test. S-HSCR: short-segment HSCR; L-HSCR: long-segment HSCR; TCA: total colonic aganglionsis; TIA: total intestinal aganglionosis.

**Table 2:** Analysis of association of allelic frequencies of SNPs rs2147555 with HSCR.

	Cases/controls (*n*)	Risk allele frequency in cases/controls	*P*_obs_	*P*_adj_	OR (95% CI)	*P*_emp_
SNP rs2147555						
Total HSCR	1469/1473	0.107/0.085	4.16 × 10^−3^	0.018	1.291 (1.084-1.538)	4.41 × 10^−3^
S-HSCR	1034/1473	0.110/0.085	0.003	0.022	1.330 (1.100-1.608)	3.12 × 10^−3^
L-HSCR	295/1473	0.111/0.085	0.044	0.086	1.344 (1.007-1.794)	0.051
TCA	82/1473	0.091/0.085	0.781	0.917	1.081 (0.626-1.867)	0.778
TIA	3/1473	0.167/0.085	0.476	0.481	2.147 (0.250-18.45)	1

*P*_obs_: unadjusted *P* values; *P*_adj_: adjusted *P* values using logistic regression analysis by including the covariate of sex; *P*_emp_: empirical *P* values obtained by performing 100,000 Monte-Carlo simulations; OR: odds ratio; CI: confidence interval.

**Table 3:** Analysis of association for genotypic frequencies of SNPs rs2147555 with HSCR under different genetic models.

	Model	*P*_obs_	*P*_emp_
SNP rs2147555			
Total HSCR	Dominant	0.011	0.012
	Recessive	0.027	0.027
	Genotypic	0.004	0.007
S-HSCR	Dominant	0.006	0.004
	Recessive	0.051	0.064
	Genotypic	0.003	0.012
L-HSCR	Dominant	0.099	0.173
	Recessive	0.019	0.039
	Genotypic	0.030	0.031

## Data Availability

The datasets generated and analyzed during the current study are available from the corresponding author on reasonable request.
